# Semirigid Ureteroscopy Therapy against Childhood Kidney Stones

**DOI:** 10.1155/2022/7771920

**Published:** 2022-08-08

**Authors:** Xiao-Nan Mu, Long-Fei Guo, Peng-Xin Wang, Long-Yang Zhang, Si-Jun Wang

**Affiliations:** ^1^Cadres Integrative Unit 2, Central Hospital Affiliated to Shandong First Medical University, Jinan, 250013 Shandong, China; ^2^Department of Urology, Central Hospital Affiliated to Shandong First Medical University, Jinan, 250013 Shandong, China; ^3^College of Basic Medicine, Jining Medical University, Jining, 272067 Shandong, China

## Abstract

**Objective:**

The purpose of the current study was to assess the effectiveness of semirigid ureterorenoscopy (URS) as first-line therapy for early childhood patients with <20 mm stones in the pelvic, middle, or upper calices.

**Methods:**

In all, 61 pediatric kidney stone patients who had flexible ureteroscopy (fURS) between January 1, 2010, and December 31, 2019, were included in this study. Before fURS, semirigid URS employed the UreTron or holmium: YAG (Ho : YAG) laser was conducted. When semirigid URS was unsuccessful, fURS was used for retrograde intrarenal surgery (RIRS). All participants were monitored clinically for a minimum of three months after each procedure.

**Results:**

The patient's mean age was 4.52 ± 1.53 years, and 52 (83.61%) participants underwent semirigid URS successfully. Mean procedural duration of semirigid URS was 36.49 ± 7.72 min. The stone-free rate after semirigid URS was 92.16% (47/51). During the postprocedural medical observation, there were no serious adverse effects.

**Conclusions:**

Based on the present study's findings, semirigid URS is a low-risk, effective therapy for kidney stones in selected pediatric patients.

## 1. Introduction

Urinary tract stone disease, after prostate disease and urinary tract infections, is the third most prevalent condition encountered by urologists. The prevalence of urolithiasis ranges from 2% to 20%, depending on a society's socioeconomic and geographic composition [1]. Although the frequency of stone disease in children is lower than in adults, it remains a severe health concern, particularly in endemic areas [2]. Pediatric stone disease causes 1%–5% of all urinary tract stone disease cases in developed countries and 30% in developing countries. The incidence of pediatric stone disease rises by 3% annually [3]. Ureteral stones smaller than 4 mm are frequently expelled gradually in children. However, bigger ureteral stones are more likely to require procedures such as shock wave lithotripsy (SWL) or ureterorenoscopy (URS) [4].

Shock wave lithotripsy (SWL) is the initial therapeutic option for kidney stones occurring during childhood since it is noninvasive. With the development in technology and the patient's request for rapid stone removal, fURS has become an ideal option for pediatric patients [5]. With the use of smaller diameter semirigid ureteroscopes and the holmium : YAG laser, endoscopic therapy for pediatric patients with upper tract stones, including pelvic kidney stones, has become efficient and safe [6, 7]. Furthermore, based on our experience, semirigid URS can approach upper and middle calyces in some pediatric patients under 7 years of age without difficulty. It is low risk and efficacious as a therapy against pediatric urolithiasis. Compared to fURS, the advantage of semirigid URS is its more significant working channel, lower cost, and less radiation exposure, and most patients do not need prestent insertion under anesthesia. This investigation evaluated medical endpoints for semirigid URS in treating selected early childhood patients with kidney stones.

## 2. Materials and Methods

From January 1, 2010, to December 31, 2019, the records of early childhood patients with kidney stones who would receive fURS were retrospectively reviewed in this study. The ethtical board committee of Central Hospital affiliated to Shandong First Medical University approved this study. The parents of the study participants signed informed consent forms.

Inclusion criteria were children <7 years old, with stones within kidney pelvis, upper or middle calices, and stone size range from 6 mm to 20 mm, with or without ureteral calculi. Exclusion criteria were pediatric kidney stones having anatomical dysmorphisms, including ureteropelvic junction obstruction (UPJO).

The demographic data and laboratory results were recorded, including 24 h urine analysis and blood chemistry study. All patients received radiology-based assessments (standard X-ray, ultrasonography, and unenhanced spiral computed tomography). Stone dimension was deemed to be the longest diameter determined through low-dose CT.

### 2.1. Surgical Technique

All surgical techniques were executed by one (of the two) surgeons (Zhang LY, Wang SJ), who were experienced in endourology. Patients were under either spinal anesthesia or general anesthesia. Antibiotics were administered during the procedure. Before semirigid URS, each patient placed a 3Fr ureteral catheter or a 0.032-inch guidewire into the ureter, passing through the ureteroscope. This was done with a pediatric semirigid ureteroscope of 6.0/7.5 Fr was used in most patients. A Wolf 8/9.8 Fr 10° semirigid ureteroscope was introduced within the ureter in 2 patients because the UreTron® (Med-Sonics Corp™, USA), with a 5 Fr semirigid probe, was used. Once the stone was visible through the semirigid ureteroscope, whether semirigid URS can treat the stone should be considered in terms of the stone position.

The UreTron with a 5 Fr semirigid probe or holmium : YAG laser was used to fragment ureteral stones. A basket was used to grasp the stone when necessary. When feasible, stones in the middle calyx were transferred onto a more optimal location within the pelvis through basketing to enhance visual accuracy throughout lithotripsy. Such stones were fragmented until dimensions were minute to the level of passing out spontaneously, or any larger fragments could be retrieved. For kidney stones that semirigid URS could not observe or stone fragments could not be broken completely, fURS would be performed to complete the procedure. A 4 Fr double J stent was inserted over the guidewire (2-4 weeks) for every patient at the end of the process.

Stone clearance was recorded postprocedure through standard abdominal radiography/ultrasonography. Overall stone-free status was deemed to be the total absence of calculous when followed up 3 months after the operation.

### 2.2. Statistical Analysis

Statistical analyses were performed through SPSS 19.0® for Windows®. Dataset outcomes reflected mean ± standard deviation.

## 3. Results

Sixty-one pediatric patients with kidney stones were included in this study.  Table 1 represents important patient information. Of all 61 cases, 37 were male, and 24 were female (male/female ratio 1.542 : 1). Thirty-four patients with single pelvis stones, 9 with upper calyx stones, 8 with middle calyx stones, 3 with multiple kidney stones, 3 with contralateral ureteral stones, 3 ipsilateral ureteral stones, and 1 with bilateral kidney stones and bilateral ureteral stones were examined. The patient's mean age was 4.52 ± 1.53 years (range: 1-7). The average size of a kidney stone was 11.10 ± 2.46 mm (6-18 mm). Before coming to our institution, 11 patients (18.03%) had unsuccessful SWL procedures in other hospitals. Semirigid URS was successfully performed in 51 patients (83.61%). The fURS was performed on 6 patients (9.84%) to complete the procedure due to the restricted maneuverability of semirigid URS. A total of 4 patients (6.56%) were placed with a double-J stent for 2-4 weeks because the ureter needed to be dilated. The mean operation time of semirigid URS was 36.49 ± 7.72 min. The 3 cases with contralateral ureteral calculi and one case of bilateral kidney stones and bilateral ureteral stones underwent a single procedure. A double-J stent was inserted within every patient postsurgery, subsequently extracted during generalized anesthesia after 2-4 weeks.  Table 2 shows surgical/postsurgical data. No severe adverse events were seen in the course of the operation. Post URS fever (*n* = 4) was managed with the conservative intravenous antibiotic.

Four children who received semirigid URS were found with a fragment of less than 4 mm at the 3 months follow-up. A total of 47 (92.16%) cases were stone-free following just one semirigid URS session on 3 months follow-up. All patients completed at least a 12-week follow-up.

## 4. Discussion

It has been reported that 2-3% of all urolithiasis incidences occur during childhood [8] Increased prevalence of pediatric patients was reported in some recent studies [9, 10]. Although the justification for such an increase remains unclear, this could be mainly linked to dietary-intake shifts, warmer climates, and alternative environmental triggers [11, 12].

The past ten years witnessed an emergence of pediatric urolithiasis cases [13, 14]. Stones > 4 mm will not typically pass spontaneously [15]. SWL has been the preferred initial treatment option against pediatric kidney stones [16]. Even though SWL remains a less invasive technique, it also has innate issues. SWL has differing success rates, with several large-scale studies describing stone-free rates ranging from 60.2% to 86.9% [17, 18], and SWL needs a longer time to achieve stone-free condition. For the cases of multiple stones, the post-SWL success rate diminished to 40% [19]. Furthermore, SWL also has some complications. Steinstrasse is an established adverse event for SWL when treating pediatric upper-tract calculi. Sayed et al. reported that steinstrasse manifested within 7% of cases having stones 1-2 cm and 12% having stones 2-3 cm after SWL [20]. Bulent et al. reported pediatric steinstrasse incidence rates post-SWL was 1.9% for stones < 1 cm^2^, 15.4% for stones 1-2 cm^2^, and 19.5% for stones > 2 cm^2^ [21].

A similar result has been reported by Madbouly et al. [22]. Repeated SWL or URS under anesthesia should be considered after the formation of steinstrasse. Goel et al. reported that approximately 40% of the patient cohort needed a minimum of four SWL procedures [23]. Muslumanoglu and colleagues investigated SWL treating urinary tract stones within 344 childhood cases. 1.9 sessions of SWL were performed per stone with an anesthesia rate of 78.5%, and the stone retreatment was 53.9% at the 3-month follow-up [24]. A recent study reported 20% remnant fragments (<5 mm) after SWL, which remains clinically concerning within pediatric cases, exacerbating risks of adverse medical endpoints [25]. Furthermore, some types of stones, such as large and cystine stones, are well known to have poor results with SWL.

With the development of technology, fURS can facilitate accessibility into pelvic/renal calices. RIRS became an option for treating kidneys of size less than 20 mm. It has been reported that 58.90% of pediatric patients need to receive a prestent insertion under anesthesia [26]. And the working channel of the flexible ureteroscope is small, allowing only laser fibers and small stone extractors. Furthermore, the expensive nature and the flexible ureteroscope are easy to be damaged will increase the concern of the costs of purchasing or repairing it. The utilization of ureteral access sheath (UAS) during the RIRS can reduce renal pressures, lower surgery duration, and ease stone-free rates. It was reported that the UAS was successfully placed in 50% of children without double-J stent placement before the UAS, and 3.08% of patients suffered from ureteral wall issues due to UAS insertion [27].

In our clinical practice, semirigid URS was routinely performed before fURS. Due to limited maneuverability and demanding access to middle and lower calyces, semirigid URS is not used in renal stones in adult patients. Because of the small collection system in children and their low body weight, miniaturized ureteroscopes and related accessories, such as the holmium : YAG laser and the UreTron, semirigid URS, have become feasible for the treatment of stones in the pelvis, upper or middle calyx in pediatric patients. During lithotripsy, we find that the stones are not as hard as they are in adults. The holmium : YAG laser has differing fiber dimensions catering to multiple cystoscope platforms, both semirigid and flexible ureteroscopes, and is versatile in fragmenting stones of all compositions [28, 29].

The stone was fragmented into pieces small enough to pass spontaneously. In our series, 49 patients received holmium : YAG laser lithotripsy. During the final phases of this investigation, 2 cases received the UreTron lithotripsy. The UreTron, an ultrasonic lithotripter with precise control probe vibration and high stone removal efficiency, was introduced recently into urology for treating urolithiasis. The UreTron needs a short learning curve because most urologists are familiar with the performance of a probe. Borofsky et al. found the UreTron could remove the stone with fast stone clearance, even in treating “hard” stones [30]. The stone fragments could become absorbed from the patient's body when the stone is fragmented into pieces. The stone-free status can be achieved earlier.

Fluoroscopy is usually used in RIRS, and the length of surgery determines the amount of radiation exposure. Children are more radiation-sensitive than adults [31]. It was reported that the median fluoroscopy time during RIRS in pediatric patients was 0.5 ~ 0.55 min [26]. Although ultrasound-guided endoscopy has been reported recently, fluoroscopy is valuable for cases with higher body mass index (BMI), congenital anomalies, and a history of previous surgeries. Fluoroscopy is still the preferred method by many physicians worldwide. No patients in our group receive radiation exposure during the operation.

In order to circumvent the increase of intrarenal pressure during the surgery, we tried to keep appropriate irrigation pressure. A 3 Fr stent was placed within the pelvis when the holmium : YAG laser lithotripter was employed. Four cases (7.84%) developed postoperative fever among patients with semirigid URS and were managed with conservative intravenous antibiotics. No life-threatening complications were observed in our study. Our complication rate was 7.84%, comparable to other recent studies [4, 32].

The routine insertion of a ureteral stent after semirigid URS was previously a standard procedure. Some children with a placed stent may feel discomforts, such as urgency, frequency, flank pain, and need removal of the stent under anesthesia. Tan et al. recommended a stent will be placed in such conditions: the procedure has been prolonged, the stone has been impacted, the ureteral orifice has been balloon dilated, and ureteral trauma is present [6]. As a urolithiasis cure center, most patients attending our institution had to cover a long distance for medical care. Within this investigation, a ureteral stent was always inserted after URL to ensure drainage efficiency and to avoid postoperative severe colic problems. No severe complications related to stent insertion were found during the operation and the follow-up in all cases, similar to Hussein and Gohar [33].

It is controversial to perform active orifices dilation before inserting the ureteroscope in children [34]. This investigation did not conduct active dilation of the ureteral orifice. Within our series, a double-J stent was inserted in four cases where semirigid URS did not enter the renal pelvis. We completed the procedure in all of these patients 2-4 weeks after the first session. In our semirigid URS-treated patients, no patient experienced chronic upper-tract dilation or UTI after treatment throughout follow-ups.

During medical observations, our series showed that the stone-free rate for semirigid URS treated cases was 92.16% (47/51). Slavkovic et al. reported that the SWL stone-free rate for treating pediatric kidney stones was 49.0% [8]. Tan et al. found a 60.2% stone-free case rate achieved post-SWL [17]. Raza and colleagues reported stone-free, approximating 84% in kidney stones < 20 mm cases [35]. It was much more favorable compared to stone-free rates within previous SWL investigations.

This investigation had limitations, such as the lack of stone analysis because of the shortage of such apparatus in our department, which remains prevalent within clinical settings due to the unidentified biochemical nature for established calculi prelithotripsy. Huang et al. reported that the predominant pediatric stone is calcium oxalate-based, whereby 60-70% of studied patients had upper-urinary tract stones [36], similar to Jallouli et al. reported [37] just as in adult patients. The other limitation is one center's experience having a relatively minute dataset.

Our investigation focused on early childhood patients with selected kidney stones who will receive fURS. Semirigid URS may be a choice if the stone can be observed and treated by semirigid URS. Semirigid URS is low-risk and effective in treating selected kidney stones. Most children become stone-free following a single session. In contrast, the performance of semirigid URS can improve lithotripsy efficiency due to its more significant working channel, lower radiation exposure, and reduced costs.

## 5. Conclusions

Semirigid URS is a low-risk and cost-effective therapy against selected early childhood renal stone patients, especially those with stones within the renal pelvis and upper and middle calices. There is an increasingly important part of URS in the future treatment of pediatric urolithiasis.

## Figures and Tables

**Table 1:** Data on the demographic and clinical features of the study participants (*n* = 61).

Variable	Number of participants (%)
Sex	
Male	37 (60.66%)
Female	24 (39.34%)
Ratio (male/female)	1.542
Clinical presentation	
Abdominal pain	39 (63.93%)
Hematuria	13 (21.31%)
UTI	9 (14.75%)
Urine parameters	
Hypercalciuria	12 (19.67%)
Hyperuricosuria	2 (3.28%)
Hyperoxaluria	0
Hypocitraturia	0
Cystinuria	0

**Table 2:** Procedural outcomes and efficacy.

Procedure	Frequency	*N* (%)
Stent insertion	4	6.56% (4/61)
Semirigid URS	51	83.61% (51/61)
Operation time (min)	36.49 ± 7.72	
*Lithotriptor*		
Holmium: YAG laser	48	94.12% (48/51)
UreTron	3	5.88% (3/51)
*Complications after semirigid URS*		
Fever	4	7.84% (4/51)
SFR after semirigid URS	47	92.16% (47/51)
FURS	6	9.84% (6/61)

## Data Availability

All data from this study are available upon request from the corresponding author.
